The article "Determining Prevalence of Anemia and Its Associated Factors in Cameroon: A Multilevel Analysis" was published in 2021. Journal: Biomed Res Int.

# Determining Prevalence of Anemia and Its Associated Factors in Cameroon: A Multilevel Analysis

**DOI:** 10.1155/2021/9912549

**Published:** 2021-11-03

**Authors:** Betregiorgis Zegeye, Bight Opoku Ahinkorah, Edward Kwabena Ameyaw, Abdul-Aziz Seidu, Mpho Keetile, Sanni Yaya

**Affiliations:** ^1^Shewarobit Field Office, HaSET Maternal and Child Health Research Program, Addis Ababa, Ethiopia; ^2^School of Public Health, Faculty of Health, University of Technology Sydney, NSW, Australia; ^3^Department of Population and Health, College of Humanities and Legal Studies, University of Cape Coast, Ghana; ^4^Population Studies and Demography, University of Botswana, Gaborone, Botswana; ^5^University of Parakou, Faculty of Medicine, Parakou, Benin

## Abstract

**Background:**

Anemia constitutes a major public health concern, which is associated with maternal and perinatal mortality. In low- and middle-income countries, the burden of anemia is profoundly high. Cameroon, as one of the low- and middle-income countries, has a disproportionate anemia burden. Factors associated with anemia prevalence are largely unknown in Cameroon. Hence, we determined the prevalence of anemia and its individual/household and community-level factors among adult women in Cameroon.

**Methods:**

We derived data from the 2018 Cameroon Demographic and Health Survey for analysis in this study. Using the Stata version 14 software, univariate multilevel logistic regression analysis was used to select variables that had significant association with anemia at *p* < 0.05. Statistically significant variables were included in a multivariable multilevel logistic regression modelling to examine their associations with anemia. Results were reported using adjusted odds ratios (AOR) with their respective 95% confidence interval (CI).

**Results:**

A total of 6,809 women aged 15-49 years were involved in this study with a mean age 30 ± 11.87 years. Approximately two-fifths of women were anemic. Of them, 0.8% were severely anemic, while 17.4% and 21.5% were moderately and mildly anemic, respectively. Current employment status (yes AOR = 0.77, 95% CI; 0.61-0.96) and parity (1-2 children AOR = 0.61, 95% CI; 0.44-0.86) were the main individual level factors associated with anemia, whereas region (Douala region AOR = 2.65, 95% CI; 1.61-4.36, North-West region AOR = 0.53, 95% CI; 0.28-0.99) was the community-level factor associated with anaemia.

**Conclusion:**

Empowerment of women through employment opportunities as well as focusing special attention in region where high prevalence of anemia could be crucial to decrease the burden of anemia and related maternal and perinatal mortality in the country.

## 1. Introduction

Anemia is a state characterized by a decrease in the level of hemoglobin in the blood that results from a reduced quality or quantity of red blood cells which reduce oxygen-carrying capacity to tissues [1, 2]. Anemia is a derivative of the multifaceted interaction of factors such as diet; communicable diseases such as malaria, HIV, and soil transmitted helminthes particularly hookworm infestation; and socio-demographic and economic factors [3].

Since anemia leads to an impaired oxygen circulation in the blood, it may lead to adverse maternal and birth outcomes, poor child growth, impaired cognitive capacity and learning ability, and reduced work productivity and income earning during adulthood [4]. As a result of the abovementioned causes, anemia in later life can lead to substantial economic loss, decrease gross domestic product (GDP), and increase treatment costs [5]. Anemia profoundly increases the likelihood of maternal and infant morbidity and mortality [6].

Anemia remains one of the major public health problems, affecting one-third of all adults and nearly two billion people globally [7–9]. Of those 56 million are pregnant women [5, 10]. Although it is prevalent among pregnant women, it occurs among women of all ages [10–12]. It has been observed that anemia impacts the lives of nearly half a billion of women in their reproductive age groups globally. Of this total, about 20.2 million women are severely anemic [13]. In low-and middle-incomecountries, the burden of anemia remains high and affects two-thirds of women in the reproductive age [14].

Since 2011, there has been a rise in maternal mortality in Cameroon, with 782 deaths/100,000 live births occurring in 2011 [15]. In furtherance, daily maternal mortality cases in the country stand at 12-13 cases [16]. This is an indication that Cameroon can be considered among sub-Saharan African countries with the highest prevalence of maternal mortality [15, 16]. Anemia is one of the causes of maternal mortality in Cameroon [16] [16]. According to USAID report, 39.5% of women of reproductive age in Cameroon were anemic in 2011. Out of these, 30.2% and 8.7% were mild and moderately anemic, while 0.6% were severely anemic [17].

Anemia among women has mostly been attributed to nutritional deficiency, specifically, iron deficiency [18]. To improve the use of iron supplementations in pregnant women, the theory of planned behavior is often recommended [19]. The theory of planned behavior was developed by Fishbein and Ajzen and is categorized into attitude, subjective norms, behavioral intention, and behavior [20]. Attitude in the theory refers to a positive or negative evaluation of behavior that is based on behavioral beliefs and an assessment of behavior outcomes and attitudes toward behavior. Subjective norms have been described as an evaluation based on the assumption that individuals are subjected to different social influences such as that from parents, a spouse, and religious leaders. Behavioral intention refers to the decision and the will of the individual to behave in a particular manner while behavior is an individual's observable response in a given situation with respect to a given target [20]. Beyond improving nutritional deficiency through education and behavioral change, several studies have found individual/household level-maternal level of education, occupation, partner's level of education and occupation, improved sanitation, contraceptive use, pregnancy termination, parity, sex of household head, media exposure, wealth quintile economic status and religion [21–25] and community-level factors such as place of residence, region [23, 26], and community literacy level and socioeconomic status [27] as predictors of anemia.

Despite the diverse predictors of anemia, most of the studies have focused on single factors, thereby not providing a holistic recognition of the factors associated with anemia among women at both the individual/household and community levels. This problem can be resolved with the use of multilevel analysis that takes into account the hierarchical levels of predictors of anemia. Again, multilevel modelling helps to take into account the household/community-level factors and how they interact with individual-level factors to predict anemia. A multilevel approach will contribute to an understanding of both the individual/household and community-level factors that predict anemia. In Cameroon, few studies related to anemia are available [28, 29]. However, their focus is on pregnant women [28, 29], covered limited area [28, 29], and facility-based as well as hematological aspects [28, 29]. To fill this gap, we were therefore motivated to investigate the individual/household and community-level factors associated with anemia among women in Cameroon.

## 2. Materials and Methods

### 2.1. Study Design

The study followed a cross-sectional study design. We used the 2018 Cameroon Demographic and Health Survey (CDHS) for the analysis. This survey was conducted by the National Institute of Statistics (NIS), in collaboration with the Ministry of Public Health [30], the United States Agency for International Development (USAID), and other national and global institutions [30], with technical and financial support of ICF International and USAID, respectively. The 2018 CDHS is aimed at providing reliable estimates of fertility levels, marriage, sexual activity, fertility preferences, family planning methods, breastfeeding practices, nutrition, childhood and maternal mortality, maternal and child health, domestic violence, malaria, and HIV/AIDS and other sexually transmitted infections (STIs) that can be used by program managers and policymakers to evaluate and improve existing programs. The sampling design applied for the 2018 CDHS was a two-stage stratified cluster sampling technique. At the first stage, a stratified sample of 469 enumeration areas (EAs) also called clusters is selected with *probability proportional to size* (PPS): in each stratum, a sample of a predetermined number of EAs is selected independently with probability proportional to the EA's measure of size. An EA is usually a geographic area that groups a number of households together for convenient counting purposes for the census. The best frame is the list of *enumeration areas* (EAs) from a recently completed population census. A complete list of EAs which covers the survey area entirely is the most ideal frame for DHS surveys. In the selected EAs, a listing procedure is performed such that all dwellings/households are listed. At the second stage, after a complete household listing is conducted in each of the selected EAs, a fixed (or variable) number of households are selected by equal probability *systematic sampling* in the selected EAs.

The total sample size for a DHS survey with a number of survey domains (design domain) is the sum of the sample sizes over all domains. An appropriate sample size for a survey domain is the minimum number of persons (e.g., women age 15-49) that achieves the desired survey precision for core indicators at the domain level. If funding is tight and fixed, the sample size is the maximum number of persons that the funding can cover. Precision at the national level is usually not a problem. In almost all cases, sample size is decided to guarantee precision at domain level with appropriate allocation of the sample.

The formula for calculating the final sample size in terms of the number of households while taking nonresponse into account is given by:

(1) $$\begin{array}{c} n={\text{Deft}}^{2}\times \frac{\left(1/P-1\right)/\alpha^{2}}{\left(R_{i}\times R_{h}\times d\right)}, \end{array}$$

where *n* is the sample size in households, Deft is the design effect (a default value of 1.5 is used for Deft if not specified), *P* is the estimated proportion, *α* is the desired relative standard error, *R*_*i*_ is the individual response rate, *R*_*h*_ is the *household gross response rate*, and *d* is the number of eligible individuals per household.

A nationally representative sample of 13,527 women aged 15-49 in all selected households and 6,978 men aged 15-64 in half of the selected households was interviewed. This represents a response rate of 98% of women and 98% of men. The sample design for the 2018 CDHS provides estimates at the national level, for urban and rural areas, and for 12 study domains. Due to security concerns, teams were not permitted to visit some zones in South-West. The data presented for that region are not representative of the region as a whole but reflect the situation in urban areas. For this reason, data from the South-West region should be interpreted with caution and should not be directly compared with data from other regions. The final report of the 2018 CDHS provides details of the methodology employed in the survey [30]. The unit of analysis in this study was women aged 15-49, and this constituted a sample size of 6,809.

### 2.2. Variable Selections and Measurement

#### 2.2.1. Outcome Variable

Anemia is the outcome variable for this study. Anemia is routinely diagnosed with a blood test. The DHS Program tests women (15-49 years) for anemia through finger prick using the HemoCue hemoglobin testing system. Testing is voluntary, and respondents receive the results of their anemia test immediately, as well as information about how to prevent anemia. Women in the reproductive age groups (15-49 years) wereoffered for anemia test. However, those women who were not tested and women whose values were not recorded are excluded from both the denominator and the numerators [31].

The measurement of anemia was done using grams per deciliter (g/dl) and was based on the level of hemoglobin concentration (Hb) in the blood [13, 32]. We included women aged 15-49 years with mild, moderate, or severe anemia or with any anemia. As mentioned by WHO, any anemia included the number of nonpregnant women whose hemoglobin count was less than 12.0 grams per deciliter (g/dl) plus the number of pregnant women whose hemoglobin count was less than 11.0 g/dl [25]. Mild anemia included the number of nonpregnant women whose hemoglobin count was between 11.0 and 11.9 g/dl plus the number of pregnant women whose hemoglobin count was between 10.0 and 10.9 g/dl. Moderate anemia included the number of nonpregnant women whose hemoglobin count was between 8.0 and 10.9 g/dl plus the number of pregnant women whose hemoglobin count was between 7.0 and 9.9 g/dl. Severe anemia included the number of nonpregnant women whose hemoglobin count was less than 8.0 plus the number of pregnant women whose hemoglobin count was less than 7.0 g/dl. At the time of creation of a recode file, an adjustment of hemoglobin count was made for altitude. Rather than change the cutoff points, the effective hemoglobin count was lowered as altitude increases, since oxygen is less available. Similarly, an adjustment is made for women who smoke [33].

#### 2.2.2. Explanatory Variables

Guided by previous literature, we considered and included numerous individual/household and community-level factors as explanatory variables for anemia among adults [21–29]. The individual/household level factors included and coded as follows: women's educational level (no education, primary, secondary, higher), husband educational level (no education, primary, secondary, higher), current employment status (no, yes), husband occupation (not working, professional or technical or managerial, clerical, sales, agricultural self-employed, service, skilled manual, unskilled manual), improved latrine (no, yes), modern contraceptive use (no, yes), ever had terminated pregnancy (no, yes), parity (no, 1-2, 3-4, 5+), sex of household head (male, female), media exposure (no, yes), wealth quintile (poorest, poorer, middle, richer, richest), and religion (catholic, protestant, other Christians, Muslim, other). Exposure to media (newspaper, radio, or television (TV)) was assessed in terms of frequency (no exposure, less than once a week, at least once a week). We coded “yes” if the respondent read newspaper or listened to radio or watched TV for at least less than once every week and “no” as otherwise. Regarding wealth index, as DHS now does not collect information on income, family wealth index was used as a proxy for monetary reputation. It is measured primarily based on element rankings generated through principal component analysis on ownership of family assets, for example, supply of drinking water, kind of toilet facility, sort of cooking fuel, and possession of television and fridge. Based on individual rankings, households have been categorized into five classes on the wealth index: poorest, poorer, middle, richer, and richest [34, 35].

The community-level factors included place of residence (urban, rural), region (Adamawa, Centre (without Yaoundé); Douala, East, Far-North, Littoral (without Dou); North, North-West, West, South, South-West, Yaoundé), community literacy level-proportion of women who can read and write (low, medium, high), and community socioeconomic status-proportion of women in the richest household quintile (low, medium-high). For community literacy, respondents who had attended higher than secondary school were assumed to be literate while all other respondents were given a sentence to read, and they were considered literate if they could read all or part of the sentence. Therefore, high literacy included respondents who had higher than secondary education or had no school/primary/secondary education and could read a whole sentence. Medium literacy were respondents that had no school/primary/secondary education and could read part of the sentence. Low literacy were respondents who had no school/primary/secondary education and could not read at all. These were categorized into appropriate tertiles where tertile 1 (lowest score, least disadvantaged) was high community literacy, tertile two (medium score) was medium community literacy, and tertile 3 (highest score, most disadvantaged) was low community literacy. For community socioeconomic status, we applied principal component analysis to calculate women who were unemployed, uneducated, and poor. A standardized rating was derived with an average rating (zero) and standard deviation [1]. The rankings were then segregated into tertile 1 (least disadvantaged), tertile 2, and tertile three (most disadvantaged) where the least rating (tertile 1) denoted greater socioeconomic status with the highest score (tertile three) denoting lower socioeconomic status.

### 2.3. Statistical Analysis

The analysis was carried out using the Stata version 14 software. Socio-demographic and other characteristics of participants were reported using frequency table. The prevalence of anemia was also presented using tables. Bivariate (univariate multilevel binary logistic regression) analysis was done to determine whether or not there are associations between each individual/household and community-level variable and anemia, and *p* value less than 0.05 was used as a cut-off point. For all variables that had significant associations during the bivariate analysis, a multicollinearity test was performed using variance inflation factor (VIF) to test the presence or absence of collinearity among them, and the result showed no evidence of multicollinearity (mean VIF = 2.69, Min VIF = 1.14, Max VIF = 5.32). After this, a two-level, multilevel logistic regression analysis was carried for all independent variables that had significant associations in the bivariate analysis. Using four steps, we carried out the multilevel logistic regression analysis using four models. The use of multilevel logistic regression was to better take into account this hierarchical data structure of the CDHS dataset which emerges by employing two-stage sampling designs. This design results in a multilevel dataset, with households, women, or men at level-1 and PSUs at level-2 [36, 37]. First, we constructed the empty/null model which represents the model that focuses on the variance in the outcome variable (anemia prevalence), attributed to the clustering at the PSUs (Model 0). Secondly, the individual/household level factors included in a model, to assess their association with prevalence of anemia (Model I). Third, we developed a model that includes only the community-level variables to assess their association with anemia (Model II). Finally, all the variables were put together to get a complete model (Model III). The multilevel logistic regression model (MLRM) consists of fixed and random effects [38–40]. The fixed effects (measures of association) demonstrate results of the association between explanatory variables and the outcome variable and were reported as adjusted odds ratios (AOR) with their 95% CIs, while the random effects (measures of variations) were assessed using Intracluster correlation (ICC) [41, 42]. Log-likelihood ratio test was used to check for model adequacy, and Akaike's Information Criteria (AIC) was used to measure how well the different models fitted the data. To cater for the complex structure of the Cameroon DHS data, we passed the “svyset” module in the model so that all the three pieces of design elements (weight, cluster, and strata) are taken into consideration. This procedure safeguards against the problem of inflated type one error and large confidence interval at the same time.

### 2.4. Ethical Consideration

For this study, we used publicly available data from DHS. DHS Program is reliable with the standards for ensuring the protection of respondents' privacy. ICF International ensures that the survey complies with the U.S. Department of Health and Human Services regulations for the respect of the right of human subjects (45 CFR 46). The IRB of National Institute of Statistics in Cameroon ensured that the survey complies with laws and norms of the nation. No further approval was required for this study since the data is secondary and available in the public domain. More details about data and ethical standards are available at http://goo.gl/ny8T6X.

## 3. Results

A total of 6,809 women aged 15-49 years were involved in this study. Of them, 1,656 (23.9%) were adolescents (within the age groups of 15-19 years) and 3,186 (45.0%) and 1,972 (27.6%) had attended secondary and primary school, respectively. Moreover, 94,129 (62.3%) of the participants were currently worked, and 1,478 (40.6%) of their husband's occupation were agricultural self-employed. Only 1,217 (17.0%) of the participants used the modern contraceptive method, and 3,878 (57.6%) had improved latrine (Table 1).

### 3.1. Anemia Prevalence across Explanatory Variables

Table 1 shows the prevalence of anemia by explanatory variables. Thus, 39.7% of women were anemic; of them, 0.8% were severely anemic, and the rest 17.4% and 21.5% were moderately and mildly anemic, respectively. The result shows that 529 (45.1%) women who had no formal education and 161 (33.7%) who had higher education had anemia. The prevalence of anemia varied based on employment status, whereby 1,567 (37.9%) women were currently working and 1,104 (41.2%) of women who did not work were anemic, respectively. There were huge variations in the prevalence of anemia across regions. For instance, the lowest prevalence (23.9%) was seen among women living in North-West region and highest prevalence (52.2%) among women living in Douala region. A higher proportion of anemia prevalence 2,259 (40.4%) was seen among women who used modern contraceptive method compared to 33.8% among women who did not use contraceptives (Table 1).

### 3.2. Correlates of Anemia

#### 3.2.1. Measure of Association (Fixed Effects) Results

As shown in Model III of Table 2, women's current employment status and parity were the significant individual level predictors, and region was the identified community-level factor that predict anemia.

Regarding the individual level factors, the odds of anemia prevalence were lower among women who were currently working (AOR = 0.77, 95% CI; 0.61-0.96) as compared to women who were not currently working. Additionally, women who ever gave birth to 1-2 children had lower odd of anemia (AOR = 0.61, 95% CI; 0.44-0.86) as compared to women who did not gave birth.

In relation to community-level factors, the odds of anemia among women who were living in Douala region were 2.7 times (AOR = 2.65, 95% CI; 1.61-4.36) higher compared to women living in the Adamawa region. However, the odds of anemia that were significantly lower among women living in North-West region (AOR = 0.53, 95% CI; 0.28-0.99) compared to women living in Adamawa region.

#### 3.2.2. Measures of Variations (Random Effects) Results

The results of the Model 0 of Table 2 show that anemia prevalence varies significantly across the clusters (*σ*2 = 0.31, 95% CI; 0.24-0.42). Model 0 revealed that 8% of anemia prevalence was linked to the between-cluster variations (ICC = 0.08). The between-cluster difference decreased from 8% in Model 0 to 7% in the model that had only the individual/household level variables (Model I). Again, the between-cluster difference decreased from 7% in Model I to 4% in the community level only model (Model II). Finally, ICC raised to 5% in the complete model (Model III) that encompassed both individual/household and community-level factors. This indicates that the differences in the probability of being anemic can be explained by the variances across the clusters.

The values of AIC confirmed a succeeding decrease, which shows that there is a considerable improvement from empty model to individual/household and community level only models and again to the complete model. This confirms the goodness of fit of the final model established in the analysis. Hence, Model III was chosen for forecasting the occurrence of anemia among women.

## 4. Discussion

Higher burden of anemia prevalence is observed in low-and middle-income countries with 89% in sub-Saharan African and Asian countries [43]. More than 38% of African women in the reproductive age group are anemic [44]. Continuous monitoring and investigating of prevalence and contextual drivers of maternal mortality causes like anemia are crucial to avert maternal and perinatal mortality especially in low-and middle-income countries such as Cameroon where the magnitude of the problem is highly prevalent.

Using the recent nationally representative 2018 Cameroon Demographic and Health Survey, we investigated the prevalence and broad-ranging individual/household and community-level predictors of anemia among Cameroonian women. Accordingly, 39.7% of women were anemic, and 0.8% were severely anemic. Also, 17.4% and 21.5% were moderately and mildly anemic, respectively. Current employment status of women and parity were the main drivers of individual/household level predictors, while region was the community-level predictor.

We found that the odds of anemia among women who had worked were lower as compared to women who did not work. Similar findings were reported in a previous study in India [45]. In low- and middle-income countries, poverty and socioeconomic status and social class within the home are the drivers for anemia especially for nutrition-related anemia in Cameroon [46]. This could be explained partly by the fact that women with job had higher confidence and freedom in accessing health care services that might later lead them to have awareness about promotion of their health [47]. This may include decisions on contraceptive use [48] that may later decrease the probability of developing anemia [49]. Women who had decision autonomy about their health care had less chance of developing anemia [50]. Having jobs is another source of income. Women who had no work might not have a chance to buy adequate foods (both in quantity and quality) or get balanced diet [51]. In Cameroon, more than 36.8% of women in the reproductive age groups had no work. Even in the participation of adult women in labor force activity is 54.5 percent, and it lowers to 38.2 percent in young women [52].

Women who had one to two delivery history had less odds of anemia compared to women who were primipara. Higher prevalence of anemia among primiparous pregnancies is mostly related to adolescence and smoking [53]. Previous study conducted in Muscat confirmed that majority (71.2%) of anemic adolescent women were below 20 years old [54]. According to WHO and study in Nepal, age and smoking behavior decrease hemoglobin concentration and lead to anemia especially among pregnant women [55]. The other explanation for less odds of anemia among women who had 1-2 delivery history could be that they might have antenatal care follow-up that is a good opportunity to contact the pregnant women with health professionals to get key information/message about prevention of anemia, through diversity and adequate intake of diet, deworming, and iron supplementation than those women who are not pregnant or delivered in the health facility.

Previous studies in Kenya [56], Ethiopia [57, 58], and Eretria [59] showed that women who had two and above ANC visits experienced good adherence with iron-folic acid supplementation and less likely to have anemia than women without ANC visit. The other justification could be that the nondelivered women had a chance of having menstrual bleeding for more periods; if so, they may have high chance to be anemic compared to women who have less period to have menstruation [60–62]. However, our finding contradicts with a previous study in Ethiopia that showed higher chance of developing anemia when parity increases due to repeated pregnancies [63]. Another study in Oman reported no association between anemia in pregnancy and parity [64].

We found substantial variation in the odds of anemia across regions. This finding is consistent with previous studies in Ethiopia [65], Rwanda [49, 66], and Tanzania [67]. The plausible justification for variation in the prevalence of anemia is that there might be the difference in socioeconomic status, cultural, and dietary patterns across regions within the same country [10]. Difference in the proportion of women who are taking iron supplementation and deworming across regions [68] and the dissimilarities of habit and cultures of eating of diversified food among societies of different regions might create dissimilarity in prevalence of anemia [69].

Additionally, the difference in the burden and management of malaria across regions might create variations in the burden of anemia [29]. Previous study in Cameroon reported that among 68.9% of anemic women in Mt. Cameroon area, 52.1% had malaria-related anemia [70]. Using the recent nationally representative survey, identifying the current individual/household and community-level factors for anemia among adult women help to design strategies that are used to reduce the burden of anemia can be considered as strength of this study. However, this study has the following limitations. First, some factors including cultural factors such as perception, beliefs, and habit of eating that need qualitative studies are not included in the study because they were not available in the dataset. Second, the cross-sectional nature of the study could not guarantee conclusion on causal-effect relationship. Finally, the findings might be affected by recall bias since some data are self-reported.

## 5. Conclusion

Nearly two-fifths of adult women in Cameroon were anemic. Women's current employment status and parity were the main individual level factors, and region was the community-level factor. Empowering women through employment opportunities as well as focusing special attention on the region where high prevalence of anemia could be the prime consideration of the Cameroon government and other stakeholders is responsible for women's health in the country.

## Figures and Tables

**Table 1:** Anemia prevalence across explanatory variables and univariate multilevel logistic regression results: evidence from 2018 Cameroon Demographic and Health Survey.

Variables	Number (weighted %)	Anemia prevalence (weighted %)	COR (95% CI)	*p* value
Women's age in years				
15-19	1,656 (23.90)	41.7	Ref	
20-24	1,246 (17.80)	39.7	0.94 (0.77-1.15)	0.581
25-29	1,205 (18.23)	36.7	0.80 (0.66-0.98)	0.033
30-34	951 (14.42)	40.4	0.90 (0.76-1.07)	0.276
35-39	757 (11.24)	42.7	0.99 (0.80-1.23)	0.976
40-44	538 (7.75)	38.3	0.86 (0.65-1.12)	0.274
45-49	456 (6.67)	36.1	0.78 (0.60-1.00)	0.059
Household head				
Male	4,982 (74.96)	40.5	Ref	
Female	1,827 (25.04)	37.6	0.89 (0.78-1.03)	0.134
Women's educational level				
No formal education	1,173 (19.93)	43.8	Ref	
Primary education	1,972 (27.60)	38.2	0.82 (0.69-0.98)	0.037
Secondary education	3,186 (45.01)	39.6	0.86 (0.72-1.03)	0.103
Higher education	478 (7.46)	35.5	0.71 (0.53-0.97)	0.033
Husband's educational level				
No formal education	706 (22.09)	45.4	Ref	
Primary education	1,260 (33.68)	35.9	0.72 (0.55-0.93)	0.014
Secondary education	1,423 (35.54)	38.6	0.80 (0.61-1.05)	0.118
Higher education	313 (8.69)	36.5	0.74 (0.51-1.06)	0.101
Current employment status				
No	2,680 (37.73)	42.5	Ref	
Yes	4,129 (62.27)	38.1	0.80 (0.70-0.91)	0.001
Husband occupation				
Not working	87 (1.93)	45.2	Ref	
Professional or technical or managerial	150 (3.74)	41.6	0.96 (0.46-1.97)	0.916
Clerical	63 (1.40)	32.3	0.60 (0.27-1.35)	0.222
Sales	662 (16.83)	36.9	0.74 (0.40-1.36)	0.346
Agricultural self employed	1,478 (40.63)	42.1	0.92 (0.51-1.67)	0.807
Service	446 (11.33)	34.1	0.66 (0.35-1.21)	0.186
Skilled manual	761 (20.55)	37.4	0.78 (0.43-1.38)	0.400
Unskilled manual	122 (3.59)	40.8	0.93 (0.42-2.05)	0.867
Improved latrine				
No	2,931 (42.40)	41.3	Ref	
Yes	3,878 (57.60)	38.6	0.87 (0.76-0.99)	0.039
Modern contraceptive use				
No	5,592 (83.00)	40.5	Ref	
Yes	1,217 (17.00)	36.2	0.89 (0.75-1.06)	0.222
Ever had termination of pregnancy				
No	5,666 (83.58)	40.1	Ref	
Yes	1,143 (16.42)	38.2	0.92 (0.78-1.09)	0.383
Media exposure				
No	2,475 (37.90)	41.1	Ref	
Yes	4,334 (62.10)	38.9	0.92 (0.80-1.04)	0.213
Wealth quintile				
Poorest	926 (16.80)	43.1	Ref	
Poorer	1,305 (18.28)	39.5	0.84 (0.67-1.04)	0.123
Middle	1,607 (20.05)	38.3	0.83 (0.66-1.04)	0.115
Richer	1,575 (22.33)	38.0	0.76 (0.60-0.96)	0.025
Richest	1,396 (22.54)	40.3	0.81 (0.64-1.03)	0.091
Religion				
Catholic	2,534 (37.93)	38.1	Ref	
Protestant	2,010 (27.07)	37.0	0.98 (0.82-1.17)	0.872
Other Christians	522 (7.14)	42.6	1.16 (0.87-1.56)	0.303
Muslim	1,529 (24.43)	43.8	1.30 (1.07-1.57)	0.006
Other	214 (3.43)	45.4	1.26 (0.92-1.72)	0.138
Parity				
No	2,040 (29.26)	42.0	Ref	
1-2	1,913 (27.57)	37.0	0.80 (0.68-0.93)	0.006
3-4	1,372 (20.56)	39.7	0.89 (0.74-1.08)	0.259
5+	1,484 (22.61)	40.1	0.88 (0.75-1.04)	0.165
Place of residence				
Urban	3,636 (54.61)	38.9	Ref	
Rural	3,173 (45.39)	40.8	1.12 (0.96-1.31)	0.128
Region				
Adamawa	491 (4.56)	44.2	Ref	
Centre (without Yaoundé)	724 (10.15)	43.4	0.97 (0.73-1.29)	0.852
Douala	559 (11.91)	53.9	1.46 (1.08-1.98)	0.012
East	596 (6.28)	32.2	0.60 (0.41-0.86)	0.007
Far-North	735 (15.49)	43.2	1.02 (0.75-1.40)	0.856
Littoral (without Douala)	459 (3.96)	45.7	1.07 (0.75-1.53)	0.683
North	663 (12.21)	39.2	0.84 (0.62-1.14)	0.284
North-West	373 (6.58)	23.7	0.38 (0.24-0.60)	0.000
West	652 (10.31)	33.8	0.63 (0.46-0.86)	0.004
South	738 (5.48)	40.4	0.86 (0.64-1.16)	0.340
South-West	183 (2.23)	35.9	0.70 (0.42-1.15)	0.163
Yaoundé	636 (10.83)	32.4	0.57 (0.40-0.83)	0.004
Community literacy level				
Low	2,315 (37.11)	40.9	Ref	
Medium	2,207 (28.95)	39.5	0.93 (0.77-1.12)	0.473
High	2,287 (33.94)	38.6	0.84 (0.69-1.01)	0.079
Community socioeconomic level				
Low	2,873 (42.78)	40.8	Ref	
Moderate	1,681 (21.34)	35.7	0.75 (0.62-0.91)	0.004
High	2,255 (35.88)	40.9	0.91 (0.76-1.10)	0.362

**Table 2:** Multilevel multivariable logistic regression results for predictors of anemia among women in Cameroon: evidence from 2018 Cameroon Demographic and Health Survey.

Variables	Model 0	Model I	Model II	Model III
Women's age				
15-19 (ref)				
20-24		1.36 (0.89-2.07)		1.36 (0.89-2.06)
25-29		1.13 (0.77-1.64)		1.10 (0.76-1.61)
30-34		1.27 (0.84-1.91)		1.21 (0.80-1.83)
35-39		1.44 (0.95-2.17)		1.38 (0.91-2.07)
40-44		1.08 (0.67-1.72)		1.03 (0.64-1.65)
45-49		1.27 (0.80-2.03)		1.24 (0.78-1.98)
Women's educational level				
No formal education (ref)				
Primary education		0.89 (0.68-1.15)		0.93 (0.72-1.21)
Secondary education		0.91 (0.65-1.25)		0.93 (0.66-1.30)
Higher education		0.73 (0.39-1.37)		0.76 (0.40-1.42)
Husband's educational level				
No formal education (ref)				
Primary education		0.87 (0.64-1.18)		0.88 (0.65-1.18)
Secondary education		1.02 (0.73-1.44)		1.01 (0.72-1.42)
Higher education		1.04 (0.64-1.69)		1.07 (0.66-1.72)
Current employment status				
No (ref)				
Yes		0.77 (0.62-0.95)^∗^		0.77 (0.61-0.96)^∗^
Improved latrine				
No (ref)				
Yes		0.89 (0.72-1.08)		0.85 (0.69-1.05)
Wealth quintile				
Poorest (ref)				
Poorer		0.93 (0.69-1.25)		0.97 (0.72-1.31)
Middle		0.82 (0.58-1.15)		0.88 (0.61-1.26)
Richer		0.85 (0.59-1.23)		0.86 (0.56-1.33)
Richest		0.88 (0.57-1.34)		0.77 (0.46-1.30)
Religion				
Catholic (ref)				
Protestant		0.98 (0.79-1.22)		1.00 (0.80-1.24)
Other Christians		1.22 (0.84-1.78)		1.24 (0.85-1.81)
Muslim		1.29 (0.98-1.70)		1.30 (0.98-1.72)
Other		1.20 (0.79-1.82)		1.14 (0.74-1.73)
Parity				
No (ref)				
1-2		0.63 (0.45-0.89)^∗^		0.61 (0.44-0.86)^∗∗^
3-4		0.79 (0.56-1.12)		0.78 (0.56-1.09)
5+		0.71 (0.50-1.01)		0.72 (0.51-1.02)
Region				
Adamawa (ref)				
Centre (without Yaoundé)			1.02 (0.77-1.35)	1.19 (0.80-1.76)
Douala			1.62 (1.16-2.27)^∗∗^	2.65 (1.61-4.36)^∗∗∗^
East			0.59 (0.42-0.85)^∗∗^	0.75 (0.46-1.23)
Far-North			0.98 (0.72-1.32)	1.25 (0.83-1.89)
Littoral (without Douala)			1.11 (0.78-1.57)	1.27 (0.77-2.09)
North			0.81 (0.60-1.10)	0.92 (0.63-1.35)
North-West			0.39 (0.25-0.61)^∗∗∗^	0.53 (0.28-0.99)^∗^
West			0.67 (0.50-0.90)^∗^	0.85 (0.56-1.29)
South			0.92 (0.68-1.24)	0.93 (0.61-1.42)
South-West			0.76 (0.46-1.26)	1.14 (0.56-2.32)
Yaoundé			0.64 (0.44-0.94)^∗^	0.89 (0.51-1.52)
Community socioeconomic level				
Low				
Moderate			0.78 (0.65-0.92)^∗∗^	0.83 (0.64-1.08)
High			0.82 (0.67-1.00)	0.92 (0.66-1.28)
Random effect result				
PSU variance (95% CI)	0.31 (0.24-0.42)	0.35 (0.23-0.51)	0.20 (0.14-0.29)	0.25 (0.16-0.38)
ICC	0.08	0.07	0.04	0.05
LR test	124.59	37.09	55.74	19.71
Wald chi-square and *p* value	Ref	*χ*2 = 47.67, *p* < 0.001	*χ*2 = 90.80, *p* < 0.001	*χ*2 = 104.62, *p* < 0.001
Model fitness				
Log-likelihood	-4488.00	-2493.54	-4443.14	-2462.53
AIC	8980.00	5041.098	8916.3	5005.06
PSU	429	429	429	429
*N*	6,809	6,809	6,809	6,809

^∗^ *p* < 0.05; ^∗∗^*p* < 0.01; ^∗∗^*p* < 0.001. Ref: reference category; AIC: Akaike Information Criterion; PSU: primary sampling unit; *N*: total observation; LR: likelihood ratio; ICC: intraclass correlation coefficient.

## Data Availability

Data for this study were sourced from Demographic and Health surveys (DHS) and available here: http://dhsprogram.com/data/available-datasets.cfm.

## Abbreviations

AIC: Akaike Information Criteria
ANC: Antenatal care
AOR: Adjusted odd ratio
CDHS: Cameroon Demographic and Health Survey
CI: Confidence interval
DHS: Demographic and Health Survey
EA: Enumeration area
ICC: Intracluster correlation
ICF: International coach federation
MLRM: Multilevel logistic regression model
PPS: Probability proportional to size
PSU: Primary sampling unit
WHO: World Health Organization.
